# A Meta-Analysis to Detect Efficacy of Physical Activity Interventions to Enhance Effects Related to the Fragility among Older Adults

**DOI:** 10.1155/2022/3424972

**Published:** 2022-08-12

**Authors:** Ping Xi, Jingyun Ding, Shandan Wan, Zixiu Zheng, Yunxiao Zhao, Xiaohua Xiao, Cong Yu

**Affiliations:** Department of Geriatric Medicine, Shenzhen Second People's Hospital, China

## Abstract

**Background:**

The role of physical activity is well-known to intercept the condition of fragility and decrease its outcomes. This study aimed to determine the efficacious physical activity intervention measure which enhances the outcomes associated to fragility in the older adults. *Material and Methods*. We searched MEDLINE, Cochrane Central Register of Controlled, and EMBASE for the published studies in the duration June 2000 to February 2020 which were further shortlisted as per the inclusion and exclusion criteria of the study. The elder population considered from the selected studies was considered in an age of 65 years or more who were pre-fragile or fragile. Here, we included the clinical as well as randomized control trials.

**Results:**

After extracting the data, we measured the risk ratio for aerobic intervention for physical intervention group as 0.55 [95% confidence interval (C.I) as 0.29, 1.03], mobility/rehabilitation interventions were nonsignificant for both groups with reported risk ratio as 1.13 (95% C.I as 0.96, 1.33), muscular strength randomized control trails as a significant integrated outcome estimate over the mobility measure, where the risk ratio was obtained as 1.17 (95% C.I 1.00, 1.35), for the randomized control trials of the mixed interventions showed a significant integrated outcome over the measures of mobility with obtained risk difference 0.03 (95% C.I -0.03, 0.09) and significant effects for daily life activities for intervention group with odds ratio 0.98 (95% C.I was 0.68, 1.41).

**Conclusion:**

From the conducted systematic review and meta-analysis, we determined a low to medium authentication that different physical activities interventions are considered to be advantageous for the pre-fragile as well as the fragile elderly people. The studies are required to be more comprehensive and clear about defining the fragility so as to assure the determination and performing of such interventions into a clinical execution.

## 1. Introduction

With the rise in the population along with the demographic variations in the maximum continental regions around the world, the health obligations of age-associated morbidity exist as a crucial health issue [1]. To conceptualize the effects of diversity of factors linked with the aging-linked results, the notion of the fragility has been put forward. As shown by the World Health Organization (WHO), the distribution of people above 60 years of age is expanding rapidly as compared to any other age range. There is a general definition associating the fragility with the increasing age and decrement of well-being [2].

As per the definition, the fragility syndrome is dependent on the existence of more than three of the given parameters: slow energy levels, decreased physical movements, weakness, poor tolerance level, and shrinking [3]. The fragility phenotype is most substantially implemented investigation in varied settings and categorizes people in three primary states: fragile, pre-fragile, and non-fragile. There are other definitions which incorporates the physiological elements like struggle with activities of daily life (ADLs), social as well as psychological dimension [4]. The elderly population with fragile conditions is at a higher risk for fall, hospital admission, and decrease in movement and death, which leads to a huge consumption of health care resources, along with an increased responsibility over the caregivers along with the unfavorable health conditions. There are evidences which reflect the association linking the regular physical actions with the upgraded muscular strength, balance, and the aerobic potential among the elderly people with fragility.

Although more of this research area that has been covered among the population with fragility has not been comprehensibly defined, the older adults with substandard mobility shall take part in exercises in a minimum three times in a week, and build up the muscular groups and rebuild and enhance the balance, thus with reduction in the risk of falls [5]. The elder population who is not able to perform exercises because of their poor state health should get involve in physical activity which is in accordance to their abilities. In spite of the comprehensive view which proposes the benefits of exercises, the signs around the exercise type, power of exercise, and timeline as well as the frequency are the most effectual characteristics for the elderly population [6].

The varied types of exercise involvements have been provided to the healthy as well as the nonhealthy elderly people. In different types of settings such as community centers, private care and residential care centers, students or professionals provide different types of support. In this study, we have conducted a systematic review and meta-analysis which targets over the physical interventions among the elderly population with pre-fragility or fragility condition so as to investigate the efficiency of the interventions to enhance the outcomes like mobility, activity of daily life, fragility, and the physical function as well as the quality of lifestyle.

## 2. Material and Methods

In this systematic review and meta-analysis, we have followed the guidelines by PRISMA, i.e., Preferred Reporting Items for Systematic Reviews and Meta-analysis. There are insignificant differences from the published procedures which were abided and the included studies were selected using the given search terms: “physical exercise,” “frail elderly,” “fragile older adults,” “functional capacity,” “randomized control trial,” “exercise,” “physical activity interventions,” “muscle strength,” “frail older adults,” and “mobility exercises.” We searched MEDLINE, Cochrane Central Register of Controlled, and EMBASE for the published studies in the duration 2000 to 2020 which were further shortlisted as per the inclusion and exclusion criteria of the study.

### 2.1. Inclusion Criteria

The studies were shortlisted for further research as per their inclusion criteria where the majority of selected studies were randomized control trials and observational studies were considered only in the case when there was no randomized controlled trials data available.

The included data like the result/outcome, intervention, and control group data were identified and these forms were further assessed. There were a total of 13 studies selected as per the inclusion criteria, and the data was labeled under the categories of the publish year of the study, country, number, age and the mean, design of the study and the duration, control type, and the intervention category.

### 2.2. Exclusion Criteria

We formed and utilized the standard forms of data extraction from the selected studies, where these forms supported as a template depending on our experience as well as proficiency.

The studies which were excluded from further research lack outcomes were wherein the age of the study population was identified less than 65 years, there was no identification of physical activity interventions, and there was either case studies or abstracts or letter or the unpublished abstracts or reported misinformation with lack of patient data. The duplicate studies or the studies which did not match the aim of the research were also excluded from further research.

### 2.3. Statistical Analysis

The meta-analysis was utilized to integrate the results obtained around all the selected studies by the results utilizing the published data from the selected data. We utilized the transition from the baseline to immediate post the intervention for both intervention as well as the control group to develop the outline of the influences in the form of standard mean difference.

This standard mean difference was utilized in the systematic review and it investigated the same result using different interventions like aerobic interventions, mobility or rehabilitation activities, muscle strengthening, and the mixed intervention activities. The standard mean difference is simplified on basis of its magnitude and for these studies the measure of variance was investigated as confidence intervals, the *p*-value or the standard error.

## 3. Results

From the total 550 identified studies, we investigated 258 full text articles which were found eligible as per the inclusion criteria of the conducted analysis. We identified and included a total of 13 studies wherein 11 were randomized control trials and 2 were clinical control trials within duration of June 2000 to February 2020 (see Figure 1).  Table 1 comprises the characteristics of the studies with further demographic data obtained from the selected studies. The effects of complete physical activity over the mobility measures were analyzed where the aerobic interventions were observed for the intervention group as shown in Table 2 and Figures 2 and 3.

### 3.1. Analyzing the Effect of Complete Physical Activity on the Mobility Measures

Aerobic interventions were found significant for intervention group with odd ratio of 0.55 (95% C.I as 0.29, 1.03) as shown in forest plot and funnel plot (Table 3 and Figures 2 and 3).

Mobility/rehabilitation interventions were nonsignificant for both groups with reported risk ratio as 1.13 (95% C.I as 0.96, 1.33) as shown in forest plot and funnel plot (Figures 4 and 5).

### 3.2. Muscular Strength Interventions

The muscular strength randomized control trails represented a significant integrated outcome estimate over the mobility measure (Table 4), where the risk ratio was obtained as 1.17 (95% C.I 1.00, 1.35) as shown in forest plot and funnel plot (Figures 6 and 7).

The randomized control trials of the mixed interventions showed a significant integrated outcome over the measures of mobility with obtained risk difference 0.03 (95% C.I -0.03, 0.09) as shown in forest plot and funnel plot (Table 5 and Figures 8 and 9).

### 3.3. Analyzing the Effect of Overall Physical Activity and Its Intervention on the Measures of Daily Life Activities

Significant effects were found for daily life activities for intervention group with odds ratio 0.98 (95% C.I was 0.68, 1.41) as shown in forest plot and funnel plot (Table 6 and Figures 10 and 11).

## 4. Discussion

This study utilized inclusion parameters of the fragility among the older adults to assess and detect a more equivalent population, although this formed more exclusion parameters which led to the exclusion of probable number of fragile population which had cases of overlapping conditions. Moreover, the range of tools as well as the interpretations implemented to outline the participants comprised of a diverse population of the study subjects. We did not assess the interventions on basis of frequency or intensity, as it was not very well outlined [19].

From the physical activity interventions, it was proposed that there was no introduction of excessive harm towards the fragile older population. There were many studies which reported no incidents of any unfavorable occurrences as well as any insignificant incidents of any physical pain, fatigue, or aches. Some studies which reported more critical occurrences were observed alike.

It was perceptible from the supervision of the selected studies that these programs should involve the expertise who possess requisite skills and knowledge like the physiotherapists, caregivers, kinesiologists, or the nurses, who are trained to execute and manage the training guidelines for such high-risk associated population of the fragile older adults. We conducted the review which helped us to identify very few studies which measured the fragility as a post-intervention result. Similarly, the extensive range of consequences implemented around the studies, comprising of the unverified tools so as to investigate the fragility, might even indicate the absence or deficiency of clarity in the fragility determination as well as detection.

There is a need of a well-formed clinical trial with definite interpretation of fragility as well as the implementation outcomes which indicate fragility determination along with detection which prevents or postpone the fragility progression among the older adults. However, a wide range of outcomes demonstrated the use of physical activity-based interventions in the clinical as well as the real-world setting, thus restricting our information over the safety and security of the interventions and inhibits the comparison of the studies.

We obtained the results immediately post the interventions that led to the long-lasting influence of the interventions which were unknown. There was analysis about the reuse of the same study subjects to contribute the data for the different measures of a given result, and this approach was preferred over the selective reporting of the influence sizes for a certain given result or the mean result measures from the same selected study to perform a standard 2-level meta-analysis. The advantage of this study was to demonstrate different physical activities interventions are considered to be advantageous for the pre-fragile as well as the fragile elderly people. The disadvantage was that there are no experiments to demonstrate this opinion. Also, the mechanism was not clarified, and further studies are needed to verify this.

## 5. Conclusion

This study demonstrated that the studies need to clearly interpret and determine the fragility in order to establish an evident recognition of older population who can be benefitted from such interventions. This would assist further development of evident guidance as well as promote the authorization and the implementation of the influential interventions into clinical exercises.

## Figures and Tables

**Figure 1:** PRISMA study over the study methods.

**Figure 2:** Forest plot of the physical activity interventions to the fragility among older adults with 95% CI was noted.

**Figure 3:** Funnel plot of the physical activity interventions to the fragility among older adults with 95% CI was noted. Mobility/rehabilitation interventions were nonsignificant for both groups with reported risk ratio as 1.13 (95% C.I as 0.96, 1.33) as shown in forest plot and funnel plot (Figures 4 and 5).

**Figure 4:** Forest plot of fragility versus non-fragility.

**Figure 5:** Funnel plot on the odds ratio of incidences of fragility versus non-fragility.

**Figure 6:** Forest plot of fragility versus non-fragility.

**Figure 7:** Funnel plot of fragility versus non-fragility.

**Figure 8:** Forest plot.

**Figure 9:** Funnel plot.

**Figure 10:** Forest plot. CI: confidence interval.

**Figure 11:** Funnel plot.

**Table 1:** Studies selected with given characteristics.

S. No.	Study	Country	Year	Number	Age + mean	Design; duration‡	Control	Delivery of intervention
1.	Kuo	Taiwan	2018	40 (81/19)	O: 67.77 I: 66.93 ± 3.91 C: 71.38 ± 4.22	Randomized control trial; 8 week	Usual care	Researcher
2.	Gill	US	2002	168 (70/30)	O: 82 I: 81.8 ± 4.0 C: 82.5 ± 4.2	Randomized control trial; 7 months	Monthly health education sessions for every individual	Physiotherapist
3.	Brown et al.	US	2000	85 (58/42)	I: 81 ± 3 C: 82 ± 1	Randomized control trial; 3 months	Home exercises	Not reported
4.	Tsang et al.	China	2013	131 (73/27§)	I: 82.33 ± 5.30 C: 83.85 ± 4.03	Randomized control trial; 12 weeks	Newspaper reading and discussion	Certified qigong instructor
5.	Chen et al.	China	2020	68 (63/37§)	I: 75.97 ± 3.19 C: 76.27 ± 6.98	Randomized control trial; 9 weeks	Usual care	Physiotherapist or community worker
6.	Yoon et al.	South Korea	2018	78 (78/22§)	O: 71.94 ± 5.27 I: 73.82 ± 3.37 C: 76.03 ± 3.27	Randomized control trial; 16 weeks	Usual care and dynamic stretching	Exercise by instructor
7.	Takatori et al.,	Japan	2016	256 (90/10)	O: 65 ± 3 I: 72.6 ± 4.1 C: 72.9 ± 5.0	Clinical controlled trial, 6 months	Lectures on health or improved activity	Physical function, mobility
8.	Faber et al.,	Netherlands	2006	277 (79/21§)	I: 86.4 ± 4.9, 83.4 ± 5.4 C: 85.9 ± 4.9	Randomized control trial; 20 weeks	Usual care	Group session by instructor
9.	Losa-Reyna et al.	Spain	2019	28(74/26§)	O: 85.2 ± 4.7 I: 83.0 ± 4.6 C: 82.4 ± 4.8	Clinical controlled trial, 6 weeks	Usual care	Not reported
10.	Liu et al., 2017	Hong Kong	2017	80(93/7††)	O: 78.32 ± 6.72 I: 78.72 ± 6.95, 75.03 ± 8.07‡‡ C: 71.90 ± 5.69	Randomized control trial; 16 weeks	Health management talks on health	Physiotherapist and instructor
11.	Kwon et al.	Japan	2015	88 (96/4††)	O: 77.8 I: 76.0 ± 6.2 C: 75.9 ± 4.9	Randomized control trial; 12 weeks	Usual health session	Certified trainer for fitness
12.	Giné-Garriga et al.	Spain	2010	50(60/40§)	I: 82.9 ± 1.8 C: 83.1 ± 2	Randomized control trial; 12 weeks	Usual health session	Physical function
13.	de Jong	Netherlands	2000	206(69/31)	O: 89.7 ± 4.6 I: 74.7 ± 3.4 C: 78.3 ± 5.6	Randomized control trial; 17 weeks	Social program	Researcher supervised

§ Value based on baseline which is not equivalent to the randomly allocated value but to the number which completed intervention I = intervention; C = control; O = overall.

**Table 2:** Aerobic intervention.

S. No.	Study	Intervention	Control	Total
1.	Kuo et al. gait	15	21	40
2.	Kuo et al. time up and go	15	21	40

**Table 3:** Mobility/rehabilitation interventions.

S. No.	Study	Intervention	Control	Total
1.	[7] gait speed	82	80	168
2.	[8] gait speed	47	33	85
3.	[9] time up and go test	41	36	131

**Table 4:** Muscle-strengthening interventions.

S. No.	Study	Intervention	Control	Total
1.	[10]; gait speed	31	32	68
2.	[11]; gait speed	21	22	78
3.	[12]; gait speed	137	71	256
4.	[1]; physical performance score (functional walking)	53	83	277

**Table 5:** Mixed interventions.

S. No.	Study	Intervention	Control	Total
1.	[13]; gait speed (usual)	9	7	28
2.	[14]; gait speed	28	20	80
3.	[15]	23	27	88
4.	[16]; gait speed (normal)	21	18	50
5.	[17]; gait speed	80	75	206

**Table 6:** Intervention.

S. No.	Study	Intervention	Control	Total
1.	[18]	15	21	40
2.	[9] LOTCA-G – memory	41	36	131
3.	[11]; Rey-15 (memory)	21	22	78

## Data Availability

The data used to support this study are available from the corresponding author upon request.
